The article "Abnormal GRHL2 Methylation Confers Malignant Progression to Acute Leukemia" was retracted in 2023. Reasons: signs of a paper mill; suspected computer-generated content; unreliable results or conclusions; concerns about the data.

# Abnormal GRHL2 Methylation Confers Malignant Progression to Acute Leukemia

**DOI:** 10.1155/2022/9708829

**Published:** 2022-07-09

**Authors:** Jing Hua, Congcong Ma, Chao Hui Wang, Yan Wang, Saran Feng, Taiwu Xiao, ChuanSheng Zhu

**Affiliations:** ^1^Department of Hematology, Shandong Provincial Qianfoshan Hospital, Shandong University, China; ^2^Department of Hematology, Liaocheng People's Hospital, Shandong University, China; ^3^Department of Hematology, Qingdao Haici Medical Group, China

## Abstract

**Purpose:**

Abnormal methylation of Grainyhead-like 2 (GRHL2) is associated with a substantial role in the malignant phenotype of tumor patients. Our present research is aimed at studying the abnormal expression of GRHL2 and the association of methylation in patients with acute leukemia and its relationship with prognosis.

**Materials and Methods:**

We used quantitative real-time polymerase chain reaction (qRT-PCR) for detecting the aberrant expression level of GRHL2 in 60 patients with acute leukemia and 60 normal controls. We analyzed the significant correlation between the expression level of GRHL2 with clinicopathological features and patients' prognosis in acute leukemia using the corresponding statistical methods. Secondly, we employed qRT-PCR and Western blotting to detect the mRNA and protein levels of GRHL2 in leukemia cell lines. Next, we used methylation-specific polymerase chain reaction (MSP) technology for detecting the methylation of GRHL2 in clinical samples with acute leukemia and cell lines. Then we investigated the demethylating effect of arsenic trioxide and 5-azacitidine on the mRNA and protein expression levels of GRHL2 in cell lines of acute leukemia. Finally, we studied the effects of arsenide trioxide and 5-azacitidine on the proliferation of leukemia cells and the TGF-*β* signaling pathway.

**Results:**

We found a lower level of GRHL2 expression not only in acute leukemia patients but also in cell lines when compared with normal controls. At the same time, the expression level of GRHL2 in patients with acute leukemia was significantly correlated with leukocyte count, platelet count, and cytogenetic risk grouping. In addition, the lower GRHL2 expression group showed a significantly lower overall survival rate in acute leukemia patients than that of patients with a higher GRHL2 expression group. Univariate and multivariate analyses revealed that the expression of GRHL2 is an independent risk factor in acute leukemia patients. The methylation level of the GRHL2 promoter region in acute leukemia patients and cell lines was significantly higher than the normal control group, and we found the elevated mRNA and protein levels of GRHL2 in acute leukemia cell lines after the use of the demethylation drug arsenic trioxide and 5-azacitidine. At the same time, arsenide trioxide and 5-azacitidine are associated with the inhibition of cellular proliferation of acute leukemia cells and also promote the elevated expression of TGF-*β* signaling pathway-linked proteins, including TGF-*β*, Smad2, Smad3, and Smad4.

The article "Abnormal GRHL2 Methylation Confers Malignant Progression to Acute Leukemia" was retracted in 2023. Reasons: signs of a paper mill; suspected computer-generated content; unreliable results or conclusions; concerns about the data.

**Conclusion:**

Increased expression and methylation level of GRHL2 are closely associated with the prognosis and malignant phenotype of acute leukemia patients and play an irreplaceable role in the occurrence and development of patients with acute leukemia.

## 1. Introduction

Acute leukemia (AL) is a critical hematological malignancy with increasing incidence year by year [1]. Its occurrence, development, and progression are a critical process involving multiple factors and steps [2]. The key molecular mechanism of the occurrence of AL has not been fully elucidated [3–5]. Epigenetics indicates the alterations of gene expression levels mediated by nongene sequence changes. It is involved in cell differentiation, maintenance of cell differentiation state, tumorigenesis, and cell senescence, mainly through DNA methylation, histone acetylation, and RNA-related silencing [6].

DNA methylation is common in hematological malignancies. Methylated DNA can prevent transcription factors from binding to it, resulting in low or no gene expression, which is an important alteration in the early initiation and development of malignant neoplastic diseases [7]. It is believed that the occurrence of leukemia is the result of genetic and epigenetic changes in protooncogene and tumor suppressor genes [8]. The tumor suppressor genes are inactivated, and the oncogenes are dominant during the formation of the tumor [9]. Leukemia cells have low genome-wide methylation and local abnormal high CpG island methylation; research shows that about 90% of the blood system of malignant tumors with at least the height of single gene methylation is closely related since this is a reversible process of genetic modification can be through to handle to restore the normal expression of gene methylation, to achieve the purpose of prevention and treatment of tumor [10].

Several studies have shown that GRHL2 showed a different degree of expression in a wide variety of tumor tissues, including epithelial squamous cell cancer, breast carcinoma, gastrointestinal cancer, liver cell cancer, colon cancer, renal carcinoma, cervical cancer, neuroblastoma, and prostate cancer. It was found that GRHL2 plays a critical role in these tumors; according to different types of tumors, it may either promote tumor growth (gastrointestinal cancer, liver cell cancer, and colon cancer) or act as a tumor suppressor (epithelial squamous cell cancer, breast carcinoma, renal carcinoma, cervical cancer, neuroblastoma, and prostate cancer) [11–14]. However, methylation of the GRHL2 gene promoter region in acute leukemia patients and leukemia cell lines remains unclear. As a new tumor suppressor gene, abnormal methylation of the GRHL2 gene promoter region may be a potential tumor molecular marker [15–17]. Therefore, this study explored the feasibility of abnormal methylation of the GRHL2 gene promoter region in patients with acute leukemia and cell lines as hematologic markers and further studied the demethylation of the GRHL2 gene by arsenide trioxide and 5-azacitidine. It is of great significance to further understand the role of DNA methylation in the development and complication of leukemia and deliver a novel theoretical basis to treat leukemia with demethylation drugs.

The article "Abnormal GRHL2 Methylation Confers Malignant Progression to Acute Leukemia" was retracted in 2023. Reasons: signs of a paper mill; suspected computer-generated content; unreliable results or conclusions; concerns about the data.

## 2. Materials and Methods

### 2.1. Object of Clinical Study

Newly treated AL patients hospitalized in Department of Hematology, Shandong Provincial Qianfoshan Hospital, Shandong University, from January 2015 to January 2020 were selected as the experimental group (*n* = 60), while healthy volunteers were collected as the normal control group (*n* = 60).

### 2.2. Inclusion Criteria and Exclusion Criteria

Inclusion criteria are as follows: (1) patients diagnosed with AL by bone marrow morphology, immunology, molecular biology, and cytogenetics according to French-American-British (FAB) standards, and their staging should be clarified; (2) complete clinical data; and (3) written informed consent signed by patients or their family members.

Exclusion criteria are as follows: (1) significant impairment of vital organ function; (2) pregnant women; (3) informed consent has not been signed; and (4) patients with incomplete follow-up data. The Ethics Committee of Qianfoshan Hospital, Shandong Province approved this study. The general clinicopathological data of acute leukemia patients are summarized in Table 1.

### 2.3. Isolation of PBMCs/BMMCs

We used Ficoll-Hypaque density gradient centrifugation (HY2015, TBD Science, Tianjin, China) to isolate peripheral blood mononuclear cells (PBMCs) and bone marrow mononuclear cells (BMMNCs) from all subjects. All collected samples were stored at -80°C.

### 2.4. Cell Line Culture

The human myeloid leukemia cell line, KG-1, was purchased from ATCC, Manassas, VA, USA, and the cell line was cultured in IMDM (Corning, NY, USA) supplemented with 20% fetal bovine serum (FBS, Gibco, Grand Island, NY), 100 U/mL penicillin, and 100 *μ*g/mL streptomycin (Sigma-Aldrich, St. Louis, MO, USA). We cultured the acute lymphoblastic leukemia cell line BALL-1 and Jurkat (Zhong Qiao Xin Zhou Biotechnology Co. Ltd. Shanghai, China) in RPMI-1640 medium which is supplemented with 10% fetal bovine serum and 1% penicillin/streptomycin in 5% CO2 at 37°C. For ensuring cellular integrity, we changed the culture medium based on standard cell culture techniques.

The article "Abnormal GRHL2 Methylation Confers Malignant Progression to Acute Leukemia" was retracted in 2023. Reasons: signs of a paper mill; suspected computer-generated content; unreliable results or conclusions; concerns about the data.

### 2.5. RNA Isolation and Quantitative Real-Time PCR (qRT-PCR)

We follow the manufacturer's instructions for extracting the Total RNA with TRIzol reagent (Thermo Fisher Scientific, Inc.). Then, we synthesized the complementary DNA (cDNA) by reverse transcription method starting with an appropriate amount of total RNA. Subsequently, we followed the instructions of the PrimeScript RT reagent kit (Vazyme Biotechnology Co., Ltd. Nanjing, CHINA) on the LightCycler 480 real-time PCR system (Roche Diagnostics, Mannheim, Germany) to perform qRT-PCR using 1 *μ*g total RNA. We employed the following reaction conditions: denaturation of Initial DNA at 95°C for 30 sec, 40 cycles of denaturation at 95°C for 5 sec, and annealing at 60°C for 30 sec. We used the comparative Cq (2^-*ΔΔ*Cq^) method for calculating the relative fold differences in this quantitative real-time PCR (qRT-PCR). We used *β*-actin as an internal control and the primer sequences are listed in Table 2. The experiment was repeated 3 times.

### 2.6. Protein Extraction and Western Blot Analyses

We washed the cells twice with cooled PBS and lysed with using RIPA and 1% PMSF (cat. no. P0013B; Beyotime Institute of Biotechnology, Beijing, China). We lysis the cells for 30 min on ice and centrifuged the mixture at 12,000 g at 4°C for 15 min. We used the BCA assay (cat. no. P0009; Beyotime Institute of Biotechnology, Beijing, China) to quantify the content of total protein based on the manufacturer's guidelines. Proteins (30 *μ*g) were served on 10% sodium dodecyl sulfate-polyacrylamide gel electrophoresis (SDS-PAGE), and then the protein was transferred on polyvinylidene difluoride (PVDF) membranes (Millipore, Billerica, MA, USA). We incubated the membranes with phosphate-buffered saline which is supplemented with 0.1% Tween-20 and 5% nonfat dry milk for blocking nonspecific binding for 1 h at room temperature. We covered the membranes with rabbit anti-human GRHL2 (1: 500, ab86611, Abcam, Cambridge, UK) and *β*-actin (1 : 1,000; #8480, Cell Signaling Technology, Inc., Danvers, MA, USA) at 4°C overnight. After one-hour incubation with horseradish peroxidase- (HRP-) conjugated goat anti-rabbit IgG antibodies (1 : 8000, Zhongshan Goldenbridge ZSGB-BIO, Beijing, China), we performed immunodetection with enhanced chemiluminescence detection kit (Millipore, Billerica, MA, USA). We used *β*-actin as a loading control. We employed the Basic Quantity One software (v4.5.0; Bio-Rad Laboratories, Inc.).

The article "Abnormal GRHL2 Methylation Confers Malignant Progression to Acute Leukemia" was retracted in 2023. Reasons: signs of a paper mill; suspected computer-generated content; unreliable results or conclusions; concerns about the data.

### 2.7. DNA Extraction, Bisulfite Treatment, and Methylation-Specific PCR (MSP)

Genomic DNA of the acute patients and acute cell lines was extracted using the DNA extraction kit (Tiangen Biotech (Beijing) CO. LTD) based on the manufacturer's guidelines. For ensuring the purity of extracted DNA, we maintained the ratio of the optical density of 260 nm to 280 nm as ~1.8. Sodium bisulfite conversion of DNA for methylation analysis was performed by the Methylation-Gold Kit (Zymo Research, Seattle, WA, USA) according to the manufacturer's instructions. For the methylated and unmethylated alleles, methylation-specific PCR (MSP) primers were designed by Wuhan Service Biotechnology Co. Ltd. (Table 3).

We determined the promoter methylation status of GRHL2 genes according to the following procedures: we used 20 *μ*L TE buffer (10 mM Tris-HCl and 1 mM EDTA; pH = 8.0) for suspending the modified DNA and quickly administered into a polymerase chain reaction (PCR) or stored at 20°C for using in future. We performed the PCR with Zymo Taq PreMix (Zymo Research). Approximately 50 ng bisulfite-modified DNA was amplified by using the MSP according to the following procedures: 95°C for 5 min; 95°C for 30 sec, 60°C (methylated) or 62°C (unmethylated) for 30 sec (45 cycles); and extension at 72°C for 5 min. We used water as a negative control. We employed the PTC 200 cycler (Bio-Rad Laboratories, Inc.) for performing the PCR. We analyze the amplified PCR products (5 *μ*L) using 2% agarose gel and visualize them under ultraviolet illumination. For each sample, we repeated MSP experiments in triplicates.

### 2.8. The Treatment of 5-Azacytidine and Arsenic Trioxide

To study the effect of epigenetic modulation, KG-1 and BALL-1 cell lines were seeded in 5 × 10^4^ cells/100 mm dishes. We collected the cells from the exponential growth phase and treated with As2O3 (0, 1.25, 2.5, and 5.0 *μ*mol/L) (Yida Pharmaceutical Co. Ltd., Harbin, China) and 5-azacitidine (0, 2.0, 5.0, and 10.0 *μ*mol/L) (Sigma, St. Louis, MO, USA)), respectively, for 48 and 72 h. We used the untreated cells as a control. We replaced the culture media every 24 hours with a fresh medium having As2O3 and 5-azacitidine. We washed the cells twice with PBS after the treatment, then centrifuged the mixture at 1000 g for 5 minutes for the next experiment.

### 2.9. MTT Assay

Cells pretreated with or without 5-azacytidine (0, 2.0, 5.0, and 10.0 *μ*mol/L), As2O3 (0, 1.25, 2.5, and 5.0 *μ*mol/L), and 5-azacytidine combined with As2O3 (2.0 + 1.25 *μ*mol/L; 5.0 + 2.5 *μ*mol/L; and 10.0 + 5.0 *μ*mol/L) were washed twice with PBS, and then resuspended in fresh RPMI-1640 supplemented with 10% FBS. To detect the effects of 5-azacytidine and arsenite on the proliferation of leukemia cell lines, 3-[4,5-dimethylthiazol-2-yl]-2,5 diphenyl tetrazolium bromide (MTT) assay (Beyotime Biotechnology, Beijing, China) was performed, 1 × 10^4^ cells/well in 200 *μ*L cell suspension was incubated for 24, 48, and 72 hours in 96-well plates, followed by addition of 10 *μ*L/well MTT reagents incubated at 37°C for 4 hours; then we removed the MTT solution and added the 150 *μ*L dimethyl sulfoxide (DMSO) for dissolving the formazan crystals. We used the BioTek ELx800 microplate photometer (BioTek ELx800, SN211805; BioTek, Winooski, VT) for measuring the spectrometric absorbance at 570 nm. All experiments were performed in triplicates.

The article "Abnormal GRHL2 Methylation Confers Malignant Progression to Acute Leukemia" was retracted in 2023. Reasons: signs of a paper mill; suspected computer-generated content; unreliable results or conclusions; concerns about the data.

### 2.10. Statistical Analysis

We employed the SPSS 25.0 software for statistical analysis. Also, we used the GraphPad Prism 8.0 software for analyzing and mapping the data. All measurement data were tested for normal distribution by the Shapiro-Wilk method. The normally distributed data were presented as mean ± standard deviation (SD) and an independent sample *t*-test was utilized to compare the mean between the two groups. In addition, the measurement data in nonnormal distribution was presented by *M* (*P*25, *P*75). We utilized the nonparametric Mann–Whitney *U* test to compare between two groups, and the nonparametric Kruskal-Wallis test was utilized to compare the multiple groups. Pearson's *χ*^2^ test was used for comparison of count data, and Fisher's exact test was used for FAB classification of acute leukemia. The Kaplan-Meier survival analysis and Cox proportional risk model were used to analyze the relationship between GRHL2 expression level and prognosis of patients with acute leukemia. *P* < 0.05 was considered the statistically significant value.

## 3. Results

### 3.1. The Expression Level of GRHL2 Is Lower in Patients with Acute Leukemia and Cell Lines

Our qRT-PCR analysis revealed that the GRHL2 expression level is significantly lower in acute leukemia when compared to the 60 patients with 60 healthy controls (Figure 1(a)). In order to further explore the correlation of GRHL2 expression with clinicopathological characteristics of acute leukemia patients, we divided the above 60 acute leukemia patients into the low-expression group of GRHL2 (above mean, *n* = 31) and the high-expression group of GRHL2 (below mean, *n* = 29) (Figure 1(b)). Subsequently, we used the Pearson Chi-square test to study the correlation of GRHL2 expression level with clinicopathological characteristics of acute leukemia patients. The findings revealed that the GRHL2 expression level is significantly correlated with leukocyte count, grouping of platelet count, and cytogenetic risk in patients with acute leukemia (Figure 1(c)); differences in gender, age, hemoglobin, bone marrow blast cell, FAB classification were not statistically significant (Table 1). Subsequently, we analyzed the expression of GRHL2 in acute leukemia cell lines (KG-1, BALL-1, and Jurkat) and normal control cell lines by QRT-PCR and Western blot. Our findings revealed that the mRNA and protein expression levels of GRHL2 in acute leukemia cell lines were significantly lower than those in the normal control group (Figures 1(d)–1(f)).

The article "Abnormal GRHL2 Methylation Confers Malignant Progression to Acute Leukemia" was retracted in 2023. Reasons: signs of a paper mill; suspected computer-generated content; unreliable results or conclusions; concerns about the data.

### 3.2. Correlation between GRHL2 Expression Level and Prognosis in Patients with Acute Leukemia

First, we utilized the Kaplan-Meier survival curve to study the relationship of GRHL2 expression level with the survival prognosis of patients with acute leukemia. Relevant results show that the lower expression group of GRHL2 showed a significantly lower overall survival rate than the patient groups with a higher level of GRHL2 expression in acute leukemia (Figure 2). These findings indicate that GRHL2 plays a substantial role in the survival prognosis of patients with acute leukemia. Then we conducted a Cox proportional risk model analysis. The results of the univariate analysis showed that hemoglobin and GRHL2 expression levels were significantly associated with the overall survival rate of acute leukemia patients. Multivariate analysis showed that the expression level of GRHL2 was an independent risk factor for the prognosis of patients with acute leukemia (Table 2).

### 3.3. Methylation Levels of GRHL2 Gene Promoter Region in Patients with Acute Leukemia and Cell Lines

We first used methylation-specific PCR to detect the methylation level of the GRHL2 gene promoter region in patients with acute leukemia and cell lines. Our investigations indicate that the GRHL2 promoter region methylation level is significantly higher in acute leukemia patients and cell lines than in the normal control group (Figures 3(a) and 3(b)). Subsequently, to investigate whether the low expression of GRHL2 in patients with acute leukemia is related to the high methylation level of the promoter region, we treated acute leukemia cell lines KG-1 and BALL-1 with the demethylation drug arsenic trioxide and 5-azacitidine. Then, qRT-PCR and Western blot were used for detecting the GRHL2 expression level in the two cell lines after treatment. We found that the mRNA and protein levels of GRHL2 in acute leukemia cell lines were significantly increased after the use of the cell demethylation drug arsenic trioxide and 5-azacitidine (Figures 3(c)–3(h)).

The article "Abnormal GRHL2 Methylation Confers Malignant Progression to Acute Leukemia" was retracted in 2023. Reasons: signs of a paper mill; suspected computer-generated content; unreliable results or conclusions; concerns about the data.

### 3.4. The Effects of 5-Azacytidine Combined with Arsenic Trioxide on the Viability of Acute Leukemia Cells

Based on the above results, we found that the demethylation drugs arsenic trioxide and 5-azacitidine could upregulate the expression of the GRHL2 by reducing the methylation level in the promoter region of GRHL2 gene in acute leukemia cell lines. In order to study whether arsenic trioxide and 5-azacitidine can inhibit the malignant phenotype of acute leukemia, we studied the effects of 5-azacytidine combined with arsenic trioxide on the viability of acute leukemia cells through an MTT experiment. The results showed that the cell viability decreased significantly after 5-azacytidine combined and arsenic trioxide treatment (Figures 4(a) and 4(b)).

### 3.5. The Effect of 5-Azacytidine Combined with Arsenic Trioxide on TGF-*β* Signaling Pathways

Related studies have shown that the activation of the TGF-*β* signaling pathway can inhibit the growth of tumor cells in most tumors. The above results showed that 5-azacytidine combined with arsenic trioxide could significantly inhibit the growth activity of acute leukemia cells. Therefore, in order to study whether the demethylation drugs arsenic trioxide and 5-azacitidine can affect the growth activity of tumor cells by regulating the TGF-*β* signaling pathway, we used qRT-PCR to study the effects of arsenic trioxide and 5-azacitidine on the TGF-*β* signaling pathway, and the results showed that arsenic trioxide and 5-azacitidine can significantly promote the expression of the TGF-*β*, Smad2, Smad3, and Smad4 (Figures 4(c)–4(f)).

## 4. Discussion

Epigenetics causes aberrant gene expression by heritable factors that do not alter the sequence of DNA itself, including DNA methylation (cytopyrimidine methylation and hydroxymethylation), histone modification, and noncoding RNA regulation [18]. DNA methylation, in particular, is a key signal that regulates gene expression during eukaryotic cell development [19]. In the tumor, researchers paid crucial attention to epigenetic regulation that critically regulates gene expression. Abnormal DNA methylation as epigenetic markers indicates a novel research avenue for the diagnosis, treatment, and prognosis of tumors [20]. At present, epigenetics is mainly monitored by DNA methylation and mRNA detection [21]. Tumor suppressor gene methylation is one of the important links in the occurrence of malignant neoplastic diseases and substantially regulates the occurrence and development of malignant neoplastic diseases [22–24]. Detection of the methylation level of specific genes is one of the important ways to monitor the evolution and outcome of malignant neoplastic diseases [25].

The article "Abnormal GRHL2 Methylation Confers Malignant Progression to Acute Leukemia" was retracted in 2023. Reasons: signs of a paper mill; suspected computer-generated content; unreliable results or conclusions; concerns about the data.

Acute leukemia is a common hematological malignancy in adults. It is characterized by abnormal clonal proliferation of immature cells in bone marrow, peripheral blood, and other affected tissues [26, 27]. With the deepening of studies on acute leukemia, epigenetics has been found to have important clinical significance in the pathogenesis of AL and has become the main direction of AL monitoring and research [28, 29]. In addition, the study of demethylation drugs has become a significant step to treat the AL, but how some regulatory genes regulate gene expression and the occurrence and development of AL remain unclear [30]. Therefore, it is of great significance to study the changes in DNA methylation and the mutations of related regulatory genes to reveal the occurrence and development of AL and to clarify the relationship between DNA methylation and regulatory genes that can provide direction for clinical treatment [31, 32].

First, the GRHL gene family has been discovered in the fruit fly *Drosophila melanogaster* [33]; there are three members of its gene family in mammals. These three members are Grainyhead-like 1 (GRHL1), Grainyhead-like 2 (GRHl2), and Grainyhead-like3 (GRHL3, [34, 35]. Besides, they are similar in sequence and biology. Studies have shown that these genes are found in various tissues, including the epidermis, urogenital tract, oral and olfactory epithelium, kidney, gastrointestinal tract, cardiovascular tissue, and lung [36]. GRHL2, the second member of this gene family, is associated with the development of the embryo, epidermal barrier formation, repairing the epidermal injury, and development of the central nervous system [37]. Furthermore, various studies revealed the deregulated expression level of GRHL2 is related to the initiation, tumorigenesis, development, progression, and prognosis of various cancers, including breast cancer, gastric cancer, colon cancer, oral squamous cell carcinoma, and liver cancer [38, 39]. In different types of tumors, GRHL2 can play different roles as either a transcriptional activator or a transcriptional suppressor. GRHL2 is highly expressed in liver cancer, breast cancer, oral squamous cell carcinoma, and other tumors, promoting tumor cell proliferation and inhibiting cell apoptosis [13, 40, 41]. On the contrary, the expression of GRHL2 is downregulated in epithelial-mesenchymal transformation- (EMT-) related breast cancers, which promoted the development of EMT [42]. Besides, it has been reported that the GRHL2 was discovered as a tumor suppressor gene because it reduces the tumor cell invasion and migration via inhibiting the TGF*β*-induced EMT in gastric cancer [43]. However, the role of GRHL2 in patients with acute leukemia remains unclear.

The article "Abnormal GRHL2 Methylation Confers Malignant Progression to Acute Leukemia" was retracted in 2023. Reasons: signs of a paper mill; suspected computer-generated content; unreliable results or conclusions; concerns about the data.

In this study, we first used qRT-PCR and Western blotting for detecting the mRNA and protein levels of GRHL2 in acute leukemia patients and cell lines and found that the GRHL2 expression level is significantly lower in patients with acute leukemia and cell lines than that in normal controls. Subsequently, we analyzed the correlation of GRHL2 expression level with clinicopathological features and prognosis of acute leukemia patients. Our results showed that the GRHL2 expression level was significantly correlated with leukocyte count, platelet count, and cytogenetic risk grouping in patients with acute leukemia. Also, the lower GRHL2 expression group showed a significantly lower overall survival rate than that of patients in the higher GRHL2 expression group. Univariate and multivariate analyses revealed that the expression level of GRHL2 is an independent risk factor for the prognosis of acute leukemia patients.

Many studies reported that the GRHL2 expression is associated with the initiation, development, progression, tumorigenesis, and survival prognosis of various cancers [41, 44], which is associated with the role of GRHL2 and aberrant promoter methylation. In the present study, we used MSP technology for detecting the methylation level of GRHL2 in acute leukemia patients, and also in cell lines. Then, we explored the effects of the demethylation drug arsenic trioxide and 5-azacitidine on the mRNA and protein levels of GRHL2 in acute leukemia cell lines. Our findings indicated that the methylation level of the GRHL2 promoter region is significantly higher in acute leukemia patients and cell lines than in the control group. Moreover, the mRNA and protein levels of the GRHL2 in acute leukemia cell lines were significantly increased after the use of the demethylation drug arsenic trioxide and 5-azacitidine. Furthermore, 5-azacytidine combined with arsenide trioxide can significantly inhibit the growth activity of acute leukemia cells.

Studies have shown that the TGF-*β*/Smads signaling pathway in normal tissues and malignant tumors have differences in expression. TGF-*β* through its signal transduction pathway and its substrate Smads protein will be biological signals from the cell membrane to the cell nucleus to activate the corresponding nucleic acid transcription to regulate cell differentiation, proliferation, adhesion, migration, apoptosis, angiogenesis, etc. [45]. In addition, the TGF-*β* signaling pathway activation is associated with the inhibition of the growth of tumor cells in most tumors [46]. In the TGF-*β*/Smads signaling pathway, Smads protein is the signal transduction molecule downstream of the TGF-*β* receptor, and its gene mutation or abnormal protein expression can lead to blocked TGF-*β* signal, the disappearance of growth inhibition, and then reduced tumor inhibition [47]. Based on this, in order to study whether the demethylation drugs arsenic trioxide and 5-azacitidine can regulate the TGF-*β* signaling pathway, thereby affecting the growth activity of tumor cells, we employed qRT-PCR for detecting the effects of arsenide trioxide and 5-azacitidine on the classical molecular markers of the TGF-*β* signaling pathway, including Smad2, Smad3, and Smad4. Our results showed that arsenide trioxide and 5-azacitidine can significantly promote the expression of TGF-*β*, Smad2, Smad3, and Smad4 [48].

The article "Abnormal GRHL2 Methylation Confers Malignant Progression to Acute Leukemia" was retracted in 2023. Reasons: signs of a paper mill; suspected computer-generated content; unreliable results or conclusions; concerns about the data.

## 5. Conclusion

In summary, we found that 5-azacytidine and arsenic trioxide restored GRHL2 expression by demethylation of the promoter region of this gene in AL cell lines and increased TGF-*β* expression and its downstream associated biomarkers, including Smad2, Smad3, and Smad4. The synergistic demethylation of 5-azacytidine and arsenic trioxide in leukemia cell lines suggests that the combination of 5-azacytidine and arsenic trioxide may have potential clinical value as demethylation drugs.

## Figures and Tables

**Figure 1:** The expression of GRHL2 in patients with acute leukemia and cell lines. (a) The expression level of GRHL2 in patients with acute leukemia. (b) The low-expression group of GRHL2 (above mean) and the high-expression group of GRHL2 (below mean). (c) The expression level of GRHL2 and clinicopathological characteristics of patients with acute leukemia. (d) The mRNA expression levels of GRHL2 in acute leukemia cell lines KG-1, BALL-1, and Jurkat. (e, f) The protein expression levels of GRHL2 in acute leukemia cell lines KG-1, BALL-1, and Jurkat.

**Figure 2:** The relationship between GRHL2 expression level and prognosis in patients with acute leukemia.

**Figure 3:** The methylation levels of GRHL2 gene promoter region in patients with acute leukemia and cell lines. (a) The methylation level of the GRHL2 promoter region in acute leukemia patients. (b) The methylation level of GRHL2 promoter region in acute leukemia cell lines. (c, d) The mRNA levels of the GRHL2 in acute leukemia cell lines after the use of the cell demethylation drug arsenic trioxide and 5-azacitidine. (e–h) The protein levels of GRHL2 in acute leukemia cell lines after the use of the cell demethylation drug arsenic trioxide and 5-azacitidine.

**Figure 4:** The effects of 5-azacytidine combined with arsenic trioxide on the viability of acute leukemia cells and the TGF-*β* signaling pathways. (a, b) The effects of 5-azacytidine combined with arsenic trioxide on the viability of acute leukemia cells. (c–f) The effect of 5-azacytidine combined with arsenic trioxide on TGF-*β* signaling pathways.

The article "Abnormal GRHL2 Methylation Confers Malignant Progression to Acute Leukemia" was retracted in 2023. Reasons: signs of a paper mill; suspected computer-generated content; unreliable results or conclusions; concerns about the data.

**Table 1:** The relationship between GRHL2 expression level and clinicopathological features in patients with acute leukemia (*n* = 60).

Characteristics	GRHL2		Chi-squared test	*P* value
	Low No. cases	High No. cases		
All patients	(*n* = 31)	(*n* = 29)		
Gender			0.577	0.448
Male	18	14		
Female	13	15		
Age (years)			0.087	0.768
≤60	14	12		
>60	17	17		
WBC count			5.668	0.017
<50 × 10^9^/L	18	8		
≥50 × 10^9^/L	13	21		
Hemoglobin (g/L)			0.243	0.622
>90 g/L	13	14		
≤90 g/L	18	15		
Platelet count (10^9^/L)			5.406	0.02
≤20 × 10^9^/L	20	10		
>20 × 10^9^/L	11	19		
Bone marrow blast cell (%)			0.276	0.599
≥30%	16	13		
<30%	15	16		
FAB classification			3.303	0.653
M0	0	1		
M1	1	3		
M2	16	12		
M3	7	6		
M4	4	3		
M5	3	4		
M6	0	0		
M7	0	0		
Cytogenetic risk group			7.601	0.022
Favorable	5	14		
Intermediate	21	13		
Unfavorable	5	2		

**Table 2:** The primers of qPCR and MSP.

Gene	Primer	Primer sequence
*GRHL2*	Forward	5′-ACAACACGGATGATGAACGA-3′
	Reverse	5′-GCATCGAACACATCGTCAGT-3′
*β-Actin*	Forward	5′-GAGCTACGAGCTGCCTGAC-3′
	Reverse	5′-GGTAGTTTCGTGGATGCCACAG-3′
*TGF-β*	Forward	5′-GGCCTTTCCTGCTTCTCATG-3′
	Reverse	5′-GAGGTCCTTGCGGAAGTCAA-3′
*Smad2*	Forward	5′-CCAGTATTAGTGCCCCGACA-3′
	Reverse	5′-TATCCAGGAGGTGGCGTTTC-3′
*Smad3*	Forward	5′-TCCATCCTGCCTTTCACTCC-3′
	Reverse	5′-CTTCTCGCACCATTTCTCCTC-3′
*Smad4*	Forward	5′-GATGACCTTCGTCGCTTATGC-3′
	Reverse	5′-GTCTAAAGGTTGTGGGTCTGC-3′
GRHL2 (MSP)-M	Forward	5′-GAAGGGTTTTATTTGAGCGCG-3′
GRHL2 (MSP)-M	Reverse	5′-ACGACCACAAATAACTTTCTCGC-3′

**Table 3:** Univariate and multivariate analysis of overall survival in patients with acute leukemia (*n* = 60).

Characteristics	Univariate analysis			Multivariate analysis		
	HR	95% CI	*P*	HR	95% CI	*P*
Gender			0.65			
Male vs. female	0.809	0.324-2.023				
Ages (years)			0.654			
≤60 vs. >60	1.282	0.434-3.787				
WBC count			0.277			
<50 × 10^9^/L vs. ≥50 × 10^9^/L	1.913	0.593-6.166				
Platelet count (10^9^/L)			0.63			
≤20 × 10^9^/L vs. >20 × 10^9^/L	1.319	0.428-4.064				
Bone marrow blast cell (%)			0.325			
≥30% vs. <30%	1.467	0.684-3.147				
FAB classification			0.42			
M0 vs. M1 vs. M2 vs. M3 vs. M4 vs. M5 vs. M6 vs. M7	1.118	0.853-1.466				
Cytogenetic risk group			0.292			
Favorable vs. intermediate vs. unfavorable	1.334	0.781-2.277				
Hemoglobin (g/L)			0.044			0.077
>90 g/L vs. ≤90 g/L	0.339	0.119-0.971		0.527	0.259-1.071	
GRHL2 expression			0.005			0.03
Low vs. high	2.836	1.373-5.860		0.331	0.159-0.689	

Abbreviations: HR: hazard ratio; CI: confidence interval.

The article "Abnormal GRHL2 Methylation Confers Malignant Progression to Acute Leukemia" was retracted in 2023. Reasons: signs of a paper mill; suspected computer-generated content; unreliable results or conclusions; concerns about the data.

## Data Availability

The data could be obtained from contacting corresponding author.
